The article "Differential Effects of Glyphosate and Roundup on Human Placental Cells and Aromatase" was published in 2005. Journal: Environ Health Perspect.

# Differential Effects of Glyphosate and Roundup on Human Placental Cells and Aromatase

**DOI:** 10.1289/ehp.7728

**Published:** 2005-02-25

**Authors:** Sophie Richard, Safa Moslemi, Herbert Sipahutar, Nora Benachour, Gilles-Eric Seralini

**Affiliations:** Laboratoire de Biochimie et Biologie Moleculaire, USC-INCRA, Université de Caen, Caen, France

**Keywords:** adjuvants, aromatase, endocrine disruption, glyphosate, herbicide, human JEG3 cells, placenta, reductase, Roundup, xenobiotic

## Abstract

Roundup is a glyphosate-based herbicide used worldwide, including on most genetically modified plants that have been designed to tolerate it. Its residues may thus enter the food chain, and glyphosate is found as a contaminant in rivers. Some agricultural workers using glyphosate have pregnancy problems, but its mechanism of action in mammals is questioned. Here we show that glyphosate is toxic to human placental JEG3 cells within 18 hr with concentrations lower than those found with agricultural use, and this effect increases with concentration and time or in the presence of Roundup adjuvants. Surprisingly, Roundup is always more toxic than its active ingredient. We tested the effects of glyphosate and Roundup at lower nontoxic concentrations on aromatase, the enzyme responsible for estrogen synthesis. The glyphosate-based herbicide disrupts aromatase activity and mRNA levels and interacts with the active site of the purified enzyme, but the effects of glyphosate are facilitated by the Roundup formulation in microsomes or in cell culture. We conclude that endocrine and toxic effects of Roundup, not just glyphosate, can be observed in mammals. We suggest that the presence of Roundup adjuvants enhances glyphosate bioavailability and/or bioaccumulation.

Glyphosate is known as the active ingredient of the broad-spectrum herbicide Roundup; it inhibits the shikimic acid pathway that is important for plant protein synthesis (Schonbrunn et al. 2001), but it has also been shown to modulate plant cytochrome P450 (Lamb et al. 1998). Glyphosate is believed to be rather specific and less toxic to the ecosystem than are other pesticides; transgenic plants tolerant to this compound have even been developed following this argument (Vollenhofer et al. 1999; Williams et al. 2000). However, mammals and humans may be exposed to herbicide residues by agricultural practices (Acquavella et al. 2004) or when they enter the food chain (Takahashi et al. 2001); glyphosate is also found as a contaminant in rivers (Cox 1998). Roundup contains acid glyphosate and adjuvants such as polyethoxylated tallowamine (Cox 1998). Its adjuvants are generally considered dilutants for regulatory purposes. Although some agricultural workers using glyphosate-based herbicides are reported to have pregnancy problems (Savitz et al. 1997), glyphosate’s mechanism of action in mammals is still questioned, and it may have several enzymatic effects (Daruich et al. 2001; Williams et al. 2000). It has also been recently shown to disrupt the animal cell cycle in urchin eggs (Marc et al. 2002) and even the post-transcriptional expression of the steroidogenic acute regulatory protein (StAR) in mouse testicular Leydig cells (Walsh et al. 2000).

In this study we tested glyphosate and Roundup toxicity on human placental JEG3 cells and also evaluated its possible capacity to act as an endocrine disruptor, as do other pesticides (Nativelle-Serpentini et al. 2003), by measuring their effects at nontoxic levels on aromatase, a mammalian cytochrome P450 enzyme crucial for sex steroid hormone synthesis. The cytochrome P450 superfamily includes numerous proteins able to metabolize xenobiotics (Nelson 1998). The enzyme aromatase is composed of the product of the *CYP19* gene (Bulun et al. 2003) and the associated nicotinamide adenosine dinucleotide phosphate (NADPH)-dependent reductase, and is responsible for the irreversible conversion of androgens into estrogens. It is considered a limiting factor involved in estrogen synthesis and thus in physiologic functions, including female and male gametogenesis (Carreau 2001), reproduction, sex differentiation, and even bone growth. It is also pharmacologically controlled in the treatment of estrogen-dependent cancers (Seralini and Moslemi 2001).

The direct action of glyphosate on aromatase could explain some effects on reproduction observed *in vivo*, at least in part; thus, we also tested glyphosate and Roundup directly on aromatase present in microsomes from human placenta and equine testis, a tissue known to be aromatase-rich (Lemazurier et al. 2001). We also purified aromatase from equine testis to assess the specificity of the interaction within the active site in this very well-characterized mammalian model (Auvray et al. 1998).

## Materials and Methods

### Chemicals.

*N*-(Phosphonomethyl)glycine (glyphosate) was purchased from Sigma-Aldrich (Saint Quentin Fallavier, France), and the pesticide Roundup (containing 360 g/L acid glyphosate; Monsanto, Anvers, Belgium) was from a commercial source. A 2% solution of Roundup and an equivalent solution of glyphosate were prepared in Eagle’s modified minimum essential medium (EMEM; Abcys, Paris, France), and the pH of glyphosate solution was adjusted to the pH of the 2% Roundup solution (~ pH 5.8). Successive dilutions were then obtained with serum-free EMEM. 3-(4,5-Dimethylthiazol-2-yl)-2,5-diphenyl tetrazolium bromide (MTT) was obtained from Sigma-Aldrich. It was prepared as a 5-mg/mL stock solution in phosphate-buffered saline, filtered through a 0.22-μm filter before use, and diluted to 1 mg/mL in serum-free EMEM. The polyclonal rabbit antibody directed against estrone (E_1_) was purchased from PARIS company (Compiègne, France). Tritiated E_1_ ([2,4,6,7-^3^H]-E_1_, 95 Ci/mmol, 3.52 TBq) was from DuPont NEN (Les Ulis, France).

### Cell line.

The human choriocarcinoma-derived placental cell line (ref JEG3, ECACC 92120308) was provided by CERDIC (Sophia-Antipolis, France). Cells were grown in phenol red–free EMEM containing 2 mM glutamine, 1% nonessential amino acids, 100 U/mL antibiotics (mix of penicillin, streptomycin, and fungizone), 1 mM sodium pyruvate, and 10% fetal calf serum (Biowhittaker, Gagny, France). Fifty thousand cells per well were grown to 80% confluence in 24-well plates, washed with serum-free EMEM, and then exposed to various concentrations of Roundup or the equivalent concentrations of glyphosate in serum-free EMEM for 1 hr or 18 hr or in serum-containing medium for longer exposures.

### MTT assay.

We used this enzymatic test, based on the cleavage of MTT into a blue-colored product (formazan) by mitochondrial enzyme succinate dehydrogenase (Mossman 1983), to evaluate JEG3 cell viability exposed to Roundup or glyphosate during various times. Cells were washed with serum-free EMEM and incubated with 250 μL MTT per well. The plates were incubated for 3 hr at 37°C, and 250 μL of 0.04 N-hydrochloric acid–containing isopropanol solution was added to each well. The plates were vigorously shaken in order to solubilize the blue formazan crystals formed. The optical density was measured using a spectrophotometer (Stratagene, Strasbourg, France) at 560 nm for test and 640 nm for reference.

### Measurement of aromatase activity in vitro by radioimmunoassay.

The conversion of androstenedione to E_1_ by the aromatase complex was measured in cell supernatants by radioimmunoassay (RIA) as previously described (Nativelle-Serpentini et al. 2003). JEG3 cells exposed to Roundup or glyphosate were washed with serum-free EMEM and incubated for 90 min with 200 nM androstenedione at 37°C in 5% CO_2_. The reaction was stopped by placing the plates on ice for 5 min, and supernatants were extracted by adding 10 volumes of diethyl ether. The extraction efficiency, evaluated by adding radio-labeled E_1_, was 60 ± 3%. The rabbit E_1_ antibody was prepared according to the manufacturer’s instructions. The sensitivity of the RIA was 10 pg/mL. Intra- and interassay coefficients of variation were 4 and 6%, respectively. The aromatase activity was expressed in relation to the protein concentration that was evaluated in cell extracts using bovine serum albumin as standard (Bradford 1976).

### RNA extraction and quantification.

Total RNA was isolated from JEG3 cells using the guanidium/phenol/chloroform method (Chomczynski and Sacchi 1987). RNA samples were treated with DNase I at 37°C for 30 min to remove genomic DNA. Then DNase I was inactivated at 65°C for 10 min.

Total RNA (1 μg) was reverse-transcribed (RT) using 100 U M-MLV-RT (Moloney murine leukemia virus reverse transcriptase) at 42°C for 45 min in the presence of 0.5 μg 18-mer oligo(dT), 500 μM of each dNTP, 50 mM Tris-HCl (pH 8.3), 75 mM KCl, 3 mM MgCl_2_, 10 mM dithiothreitol (DTT), and 6 U RNasin in a total volume of 25 μL. The absence of DNA contamination in the RNA samples was checked in controls without M-MLV-RT.

For each run, a master mix was prepared with 1 × SYBR Green buffer containing 5 mM MgCl_2_; 200 mM dATP, dCTP, and dGTP; 400 mM dUTP; 1.25 U AmpliTaq Gold DNA polymerase (Applied Biosystems, Courtaboeuf, France); and 300 nM of each primer: EXIIc sense primer, 5′ TGA GGT CAA GGA ACA CAA GA 3′, exon II specific (positions 9–28); and EXIII antisense primer, 5′ ATC CAC AGG AAT CTG CCG TG 3′, for exon III (positions 211–230) (Corbin et al. 1988). Five microliters of each diluted RT sample were added to 20 μL of the polymerase chain reaction (PCR) master mix. The thermal cycling conditions consisted of an initial denaturation step at 95°C for 10 min and 40 cycles at 95°C for 15 sec and 60°C for 1 min. We also quantified the transcripts of the housekeeping gene glyceraldehyde-3-phosphate dehydrogenase (GAPDH) as an endogenous control to normalize each sample using sense and antisense primers, 5′ CCA TCA CCA TCT TCC AGG AGC 3′ (positions 278–298) and 5′ GGA TGA TGT TCT GGA GAG CC 3′ (positions 663–682), respectively (Tokunaga et al. 1987). All PCR reactions were performed using an ABI Prism 7000 Sequence Detection System (Applied Biosystems).

### Preparation of microsomes.

Microsomal fractions (endoplasmic reticulum) were obtained from full-term placentas of young healthy and nonsmoking women (Centre Hospitalier Régional de Caen, France) and equine testis by differential centrifugations (Moslemi et al. 1997). Briefly, tissues were washed with 0.5 M KCl, homogenized in 50 mM phosphate buffer (pH 7.4) containing 0.25 M sucrose and 1 mM DTT, and centrifuged at 20,000*g*. The supernatant was then ultracentrifuged at 100,000*g*, and the final pellet was washed twice, dissolved in the same buffer containing 20% glycerol, and stored at −70°C until use. All steps of the preparation were carried out at 4°C.

### Measurement of microsomal aromatase activity.

Microsomal aromatase activity was evaluated by tritiated water release from radio-labeled substrate [1β-^3^H]-androstenedione as previously described (Moslemi et al. 1993, 1997). This method is based on the stereo-specific release of 1β-hydrogen from the androstenedione substrate, which forms tritiated water during aromatization (Dintinger et al. 1989; Thompson and Siiteri 1974). Human placental microsomes (50 μg protein) were incubated with radiolabeled androstenedione (100 pmol/tube) at 37°C for 15 min, in the presence or absence of various concentrations of Roundup or glyphosate in 1 mL total volume of 50 mM Tris-maleate buffer (pH 7.4). The reaction was started by adding 100 μL of 0.6 mM H^+^-NADPH and stopped with 1.5 mL chloroform, and then centrifuged at 2,700*g* at 4°C for 5 min. After adding 0.5 mL 7% charcoal/1.5% dextran T-70 solution into the preparation, the centrifugation was repeated for 10 min. Aromatase activity was determined by measuring the radioactivity of the 0.5 mL aqueous phase. The kinetic parameters were determined by incubating equine testicular microsomes (2 μg protein) with various concentrations of radiolabeled androstenedione in the presence of various concentrations of Roundup in 0.5 mL of H^+^-NADPH containing Tris-maleate buffer (pH 7.4) at 25°C for 3 min.

### Purification of aromatase moieties.

Reductase was obtained after chromatographic separation, by ω-aminohexyl-Sepharose 4B and adenosine 2′,5′-diphosphate agarose, respectively; hydrophobic interaction; and affinity columns (Vibet et al. 1990). The cytochrome P450 aromatase was purified from equine microsomes, after its separation from reductase, by successive chromatographic steps: concanavalin A-Sepharose 4B affinity column, diethyl amino ethyl-Sepharose CL-6B ion exchange, and hydroxyapatite-Sepharose 4B adsorption/partition columns (Moslemi et al. 1997). Protein concentration was determined as previously described (Bradford 1976).

### Measurement of reductase activity.

Reductase activity was determined by the measurement of the increasing absorbance of the preparation, corresponding to the reduction of the cytochrome C in the presence of H^+^-NADPH (Vibet et al. 1990) at 550 nm for 2 min at 37°C using a Kontron-Uvikon 860 spectrophotometer (Kontron Instruments S.A., St. Quentin Yvelines, France). The pH of the preparation was adjusted when adjusted to 7.4 by adding an appropriate volume of 10 N NaOH. After equilibration, the reaction was started by adding cytochrome C.

### Spectral studies.

The absorbance of purified equine aromatase in the presence or absence of glyphosate or Roundup was recorded from 375 to 475 nm with a spectrophotometer as previously described (Moslemi and Seralini 1997). Briefly, absorption spectra of 362 μg aromatase protein in 1.5 mL 50 mM Tris-maleate containing 2 μM androstenedione were recorded during incubation at 37°C, after adding 0.0046% glyphosate or 0.1% Roundup. The spectra of aromatase with glyphosate or Roundup alone were subtracted from the incubation spectrum.

### Statistical analysis.

All data are presented as the mean ± SE. The experiments were repeated three times in triplicate unless otherwise indicated. Statistically significant differences were determined by a Student *t*-test using significance levels of 0.01 and 0.05.

## Results

### Cell viability.

The recommended agricultural use for Roundup is 1–2% in water, so we tested its effect on human placental JEG3 cell viability at concentrations of up to 2% after 18-, 24-, or 48-hr exposures in serum-containing medium, by the MTT assay in conditions previously described (Nativelle-Serpentini et al. 2003), compared with glyphosate. The Roundup dilutions and equivalent quantities of glyphosate were adjusted to the same pH to facilitate the comparisons. The toxicity increased with time (8-fold at 0.8% between 24 and 48 hr), and the median lethal dose (LD_50_) was approximately 1.8 times lower for Roundup (0.7%) than for glyphosate (Figure 1). This difference was even visible after 1 hr of incubation in serum-free medium (Figure 2A) and increased 3-fold after 18 hr of incubation (Figure 2B). Acidity of the 2% Roundup or glyphosate solution (pH 5.80 ± 0.08 instead of pH 7.91 ± 0.16) reduced cell viability only 23% after 18 hr, and thus could not alone explain the 90% reduction of cell viability observed at this concentration. When only 0.1% Roundup was added to glyphosate, bringing small amounts of the adjuvants to the solution, the cell viability was diminished significantly (Figure 2B).

### Aromatase activity in cell culture.

We measured aromatase activity after incubation of cells in the presence of nontoxic concentrations of Roundup or glyphosate, by RIA of E_1_ formed from 200 nM androstenedione, as previously described (Nativelle-Serpentini et al. 2003). As shown in Figure 3A, after 1 hr of incubation, the estrogen synthesis was enhanced by about 40% but only with Roundup. After 18 hr of incubation, we noted a clear inhibition of aromatase activity *in vitro*, with a median inhibiting concentration (IC_50_) of 0.04% again with Roundup only. This inhibition of aromatase activity is, at least in part, assumed to be an effect on aromatase gene expression, because mRNA levels were decreased (Figure 3B). Glyphosate was inefficient alone in these conditions. But it inhibited aromatase activity with minute dilutions of Roundup, bringing adjuvants in the solution (Figure 4).

### Aromatase activity in microsomes.

We evaluated microsomal aromatase activity by tritiated water release from the radiolabeled substrate (Dintinger et al. 1989; Thompson and Siiteri 1974) in human (Figure 5) and equine microsomes. Aromatase inhibition by Roundup was equivalent in these two mammalian models. The IC_50_ was 0.6% for Roundup in these conditions and more than three times greater for glyphosate. The kinetic parameters were determined by incubating equine testicular microsomes with various concentrations of radiolabeled androstenedione and Roundup. The inhibition constant *K*_i_ (0.6%) showed a competitive inhibition (Figure 6A).

### Enzymatic activity of purified enzymes.

We further purified the enzyme moieties from the aromatase-rich equine testis, giving better yields than placenta. The incubation with the herbicide demonstrated a direct interaction of glyphosate within the active site. We obtained spectral interactions between Roundup or glyphosate and the active site of the purified cytochrome P450 aromatase by measuring the absorbance of the preparations from 375 to 475 nm. A type II spectrum was observed (Figure 6B); it was characteristic of an interaction between a nitrogen atom of the molecule and the heme iron of the cytochrome. In addition, we tested the effect of the herbicide on the ubiquitous moiety of the aromatase, which is the electron donor reductase. NADPH-dependent reductase activity was determined by the measurement of the increasing absorbance of the preparation, corresponding to the reduction of the cytochrome C. Reductase is also directly affected after purification and incubation with Roundup, but to a lesser extent (IC_50_ 5%) than the cytochrome P450 aromatase responsible for steroid binding and catalysis (Figure 7).

## Discussion

This study demonstrates that Roundup reduces JEG3 cell viability at least twice more efficiently than glyphosate. This effect increased with time and was obtained with concentrations of Roundup 10 times lower than that of the agricultural use. The presence of serum buffers the toxic effect of the herbicide. It is generally recognized that serum proteins can bind to chemicals and reduce their availability to cells. Seibert et al. (2002) have shown that the presence of albumin influences the cytotoxicity of compounds. Moreover, the lack of growth factors in serum-free medium, for instance, could also play a role in this phenomenon. In our experiments, the incubation in serum-free medium was interesting to optimize the visible effects of the compounds in the shortest time. These were also observed anyway after 48 hr in the presence of serum. The physiologic significance of these effects can be questioned, in regard to the concentration used. However, the time of exposure to pollutants may be longer *in vivo*, and here *in vitro* we observed that long times of exposure allowed low concentrations to present toxic effects. This phenomenon could be caused by metabolism, genomic action, and/or bioaccumulation of some products of Roundup. For instance, Peluso et al. (1998) demonstrated the formation of covalent links between DNA and some Roundup adjuvants. Their genotoxicity or toxicity was also noticed (Lioi et al. 1998; Mitchell et al. 1987; Vigfusson and Vyse 1980). Even though absorbed Roundup is excreted rapidly from the body, usually in feces (Brewster et al. 1991; Williams et al. 2000), a part may be retained or conjugated with other compounds that can stimulate biochemical and physiologic responses. The bioaccumulation of some of its residues may be hypothesized. For example, the harmful effect of glyphosate on semen quality after 6 weeks of post-treatment period in rabbits (Yousef et al. 1995) may be considered an indication of its retention and conjugation in the body, helped by Roundup adjuvants.

Additionally, in this work Roundup presents a differential time effect at nontoxic levels on aromatase activity of JEG3 cells; this phenomenon was already observed with other xenobiotics such as lindane and bisphenol A (Nativelle-Serpentini et al. 2003). The 40% rise in aromatase activity after 1 hr of incubation is perhaps caused by an increase of the membrane fluidity and androgenic substrate bioavailability in a first step provoked by adjuvants. By contrast, once well entered into cells, Roundup always reduced aromatase activity. Furthermore, this was associated with the decrease of *CYP19* mRNAs. Walsh et al. (2000) showed that Roundup preferentially diminished the expression of StAR mRNA by decreasing at least the rate of gene transcription.

The direct inhibition of aromatase activity by Roundup was verified in human and equine microsomes, two mammalian aromatase models that we have precisely characterized, in order to understand the active site configuration of this membrane-bound cytochrome P450 (Auvray et al. 1998; Moslemi and Seralini 1997; Seralini et al. 2003). Contrary to results obtained in cells, glyphosate had an inhibitory effect on aromatase activity in human and equine microsomes, but four times lower than the effects of Roundup. Moreover, Roundup inhibited aromatase better in cells than in microsomes (IC_50_ values, 0.04 and 0.6%, respectively). This could be explained by the difference in incubation duration (18 hr vs. 15 min) inducing metabolism and genomic action. Glyphosate penetration through the cell membrane and subsequent intracellular action appeared in our work to be greatly facilitated by adjuvants, as in plants (Haefs et al. 2002) or in animal cells, where it can act at the level of cycle regulation (Marc et al. 2002). Indeed, in this work, minute dilutions of Roundup bringing adjuvants to cells allowed the aromatase inhibitory effect of glyphosate as well as cytotoxic effects.

Moreover, the presence of Roundup in the incubation medium resulted not only in the decrease of the activity of the cytochrome P450 aromatase, but also to a lesser extent in a partial inhibition of its associated reductase. This is confirmed by kinetic and spectral studies that showed that Roundup inhibits the enzyme at the active site level in a competitive manner. Furthermore, our spectral study shows a type II spectrum for purified equine aromatase in the presence of glyphosate or Roundup at the saturating concentration of androstenedione. After androstenedione elimination, Roundup induces a type I spectrum. A type II spectrum with minimal absorbance at 390 nm and maximal absorbance at 420 nm is considered specific for an interaction between a nitrogen atom of the molecule and the heme iron of the cytochrome, whereas a type I spectrum (inverted absorbance) is observed when this type of interaction is absent. Androstenedione, a natural hormone, thus appears to facilitate pesticide access to the active site of the enzyme. However, this occurs more easily with glyphosate directly in contact with the solubilized enzyme than with Roundup, because less concentration of the former was needed to produce the same spectrum.

## Conclusion

Our studies show that glyphosate acts as a disruptor of mammalian cytochrome P450 aromatase activity from concentrations 100 times lower than the recommended use in agriculture; this is noticeable on human placental cells after only 18 hr, and it can also affect aromatase gene expression. It also partially disrupts the ubiquitous reductase activity but at higher concentrations. Its effects are allowed and amplified by at least 0.02% of the adjuvants present in Roundup, known to facilitate cell penetration, and this should be carefully taken into account in pesticide evaluation. The dilution of glyphosate in Roundup formulation may multiply its endocrine effect. Roundup may be thus considered as a potential endocrine disruptor. Moreover, at higher doses still below the classical agricultural dilutions, its toxicity on placental cells could induce some reproduction problems.

## Figures and Tables

**Figure 1:** Effects of Roundup (*A*) and equivalent quantities of glyphosate (*B*) on JEG3 placental cell viability in a serum-containing medium. This was evaluated by the MTT assay, the results are presented as percentages compared with nontreated cells. Cells were incubated with increasing concentrations of Roundup or equivalent concentrations of glyphosate for 18, 24, or 48 hr (*n* = 9). The LD_50_ is indicated by a dashed line. Error bars indicate SE.
*p < 0.05;
**p < 0.01.

**Figure 2:** Effects of Roundup and equivalent quantities of glyphosate on JEG3 placental cell viability in serum-free medium. The incubation was for 1 hr (*A*) or 18 hr (*B*). The addition of 0.02 or 0.1% Roundup shows adjuvant effects (*n* = 9). Error bars indicate SE. 
**p < 0.01.

**Figure 3:** Effects of Roundup and equivalent quantities of glyphosate on JEG3 aromatase activity and mRNA levels in a serum-free medium. Aromatase activity (*A*) was obtained with nontoxic concentrations of Roundup or glyphosate for 1 and 18 hr (*n* = 9). (*B*) Cytochrome P450 aromatase mRNA levels, normalized with GAPDH levels, in the presence of Roundup or glyphosate after 18 hr (*n* = 4). Error bars indicate SE. 
**p < 0.01.

**Figure 4:** Combined effects of glyphosate and minute levels of Roundup on JEG3 aromatase activity in serum-free medium (*n* = 9). It was obtained at non-toxic concentrations after 18 hr exposure. 
**p < 0.01.

**Figure 5:** Effects of Roundup and equivalent quantities of glyphosate on microsomal aromatase activity. Human placental microsomes were incubated with Roundup or glyphosate at 37°C for 15 min (*n* = 9). The IC_50_ is indicated by a dashed line. Similar results were obtained with equine testicular microsomes. Error bars indicate SE. 
**p < 0.01.

**Figure 6:** Kinetic and spectral studies of aromatase in the presence of Roundup or glyphosate. (*A*) Lineweaver-Burk representation of equine testicular microsomal aromatase activity in the presence of Roundup at 25°C with radiolabeled androstenedione. Comparable results were obtained with human placental microsomes (*n* = 9). (*B*) Spectral analysis of interactions between the active site of purified equine cytochrome P450 aromatase and 0.1% Roundup (left) or 0.0045% glyphosate (right). Type II spectra were obtained with Roundup or glyphosate in the presence of 2 μM androstenedione, and a type I spectrum was obtained in its absence. The results are representative of three experiments. Error bars indicate SE.

**Figure 7:** Effect of Roundup on reductase activity. Activity of purified equine reductase was measured in the presence of increasing concentrations of Roundup in nonadjusted or adjusted pH (7.4) medium for 15 min at 37°C (*n* = 9). Error bars indicate SE.
